The article "Research on Vibration Reduction Method of Nonpneumatic Tire Spoke Based on the Mechanical Properties of Domestic cat's Paw Pads" was published in 2021. Journal: Appl Bionics Biomech.

# Research on Vibration Reduction Method of Nonpneumatic Tire Spoke Based on the Mechanical Properties of Domestic cat's Paw Pads

**DOI:** 10.1155/2021/9976488

**Published:** 2021-05-16

**Authors:** Haichao Zhou, Huiyun Li, Ye Mei, Guolin Wang, Congzhen Liu, Lingxin Zhang

**Affiliations:** ^1^School of Automotive and Traffic Engineering, Jiangsu University, Zhenjiang 212013, China; ^2^School of Transportation and Vehicle Engineering, Shandong University of Technology, Zibo 255000, China; ^3^AEOLUS Tyre Co. Ltd., Jiaozuo 454003, China

## Abstract

Although there is no risk of puncture, the vibration problem caused by discontinuous structures limits nonpneumatic tire development (NPT). The vibration reduction of nonpneumatic tires is a solvable urgent problem. This current study analyzed the dynamic grounding characteristics and the vibration reduction mechanism of the cat's paw pads and then applied the mechanical properties to the bionic design of nonpneumatic tire spokes to solve the vibration problem. Domestic cats' paw pads' dynamic grounding characteristics were determined using the pressure-sensitive walkway, high-speed camera, and VIC-2D. The results indicated that the mechanical characteristics of swing deformation of paw pads during the grounding process attenuated the grounding stress and buffered the energy storage to achieve the vibration reduction effect. According to the similarity transformation, a finite element model of NPT that could accurately reconstruct the structure and realistically reflect the load deformation was employed. The structure design of asymmetric arcs on the spokes' side edges was proposed, and it can effectively reduce the radial excitation force of NPT. The three parameters, the asymmetric arc, the thickness, and the curvature of spokes, were used as design variables to maximize the vibration reduction. The orthogonal experimental, the Kriging approximate model, and the genetic algorithm were carefully selected for optimal solutions. Compared with the original tire, the results showed that peak amplitude 1, peak amplitude 2, and the root square of the optimized tire's amplitudes were reduced by 76.07%, 52.88%, and 51.65%, respectively. These research results offer great potential guidance in the design of low-vibration NPT.

## 1. Introduction

As the only direct contact medium between the vehicle and the road, the tire directly affects the steering stability, driving the vehicle's safety and riding comfort. However, traditional pneumatic tires have safety hazards such as punctures and air leaks, which seriously affect safe vehicle driving [1]. Therefore, nonpneumatic tires (NPT) have demonstrated development advantages regarding safety, economy, environmental protection, and wear resistance [2]. Since the advent of Michelin's Tweel tire [3], a variety of nonpneumatic tires such as the Air Free Concept launched by Bridgestone have emerged [4]. These include the honeycomb structure tires which are jointly developed by Resilient Technologies and the University of Wisconsin-Madison Polymer Engineering Center [5] and i-Flex nonpneumatic safety tire designed by Hankook [6]. Similarly, “N-wheel” nonpneumatic tire with negative Poisson's ratio spoke structure was developed by Tianqu Non-Pneumatic Wheel Technology Co., Ltd. and BAIC Group [7]. Mechanical elastic wheel was also proposed by Zhao Youqun of Nanjing University of Aeronautics and Astronautics [8, 9]. And nonpneumatic tires with different support structures such as truss, octagonal and gradient elasticity [10–12] are but few of the evolution in nonpneumatic tire research, design, and development.

The article "Research on Vibration Reduction Method of Nonpneumatic Tire Spoke Based on the Mechanical Properties of Domestic cat's Paw Pads" was published in 2021. Journal: Appl Bionics Biomech.

Peculiar to all these innovations is a prominent vibration problem associated with nonpneumatic tires, which limits the speed of vehicles running on nonpneumatic tires. This remains a challenge in the development of nonpneumatic tires. Consequently, vibration reduction has become one of the key areas of improvement in the development of nonpneumatic tires. Compared with the better uniformity of mass distribution of pneumatic tires, the discontinuous support structures of nonpneumatic tires introduce nonuniform mass distribution, causing nonuniform stiffness that results in a local vibration effect [13–15]. As a replacement for pneumatic tires' air pressure, the nonpneumatic tires' spokes play the role of supporting, cushioning, damping, and providing force [16, 17]. Hence, this has made the design of spokes a key focus of various studies on nonpneumatic tires. Manga [18] found that the spoke vibration was not a forced vibration related to the rolling speed but a resonance excited by the buckling and rebound phenomena when the spoke entered and left the contact zone. Bezgam [19] obtained the contribution of spoke shape parameters to spoke vibration through orthogonal experiment, adjusted the thickness and curvature of adjacent spoke pairs based on this, and proposed the design concept of alternate spoke pairs to reduce the amplitudes of spokes and ground vibration. Proddaturi [20] proved in his research that the spokes' length and curvature have the greatest influence on vibration, followed by the thickness of the shear beam, the thickness of spokes, and the number of spokes. The thickness of the inner and outer coverages and the inner and outer DeRad were reported to have less influence. When adjusting the shear modulus of the spokes, Narasimhan [21] concluded that the change of the material led to the change of stiffness, and the increase of the stiffness caused the spoke vibration to decrease. Meanwhile, the spoke material's change had a greater impact on the spoke vibration than the shear band material's change.

The article "Research on Vibration Reduction Method of Nonpneumatic Tire Spoke Based on the Mechanical Properties of Domestic cat's Paw Pads" was published in 2021. Journal: Appl Bionics Biomech.

In the long-term evolution of animals, a variety of biological structures and functional characteristics highly adaptable to nature have been formed. Researchers use these principles to invent and innovate technologies. For example, Romano et al. [22] found in the study of the escape direction of Locusta migratoria a high plasticity of those escape motor outputs that are occurring almost in real time with the perceived stimuli, making them greatly adaptable and compliant to environmental changes, to be effective and reliable. The locust's strong jumping ability allows it to avoid predators and start flying, and the combined action of the rigid claws and the adhesive pads ensures that the static contact between tarsus and ground, which can achieve a smooth jump on a smooth surface; in addition, the large take-off angles also allow locusts to achieve better performance on smooth surfaces, which provides inspiration for the jumping robot design [23]. When catching prey, cats need to have a strong ability to reduce vibration, so as to weaken the impact from the ground and achieve characteristic silence. As the only body part in contact with the ground, the paw pads play an important role in vibration reduction realization. Mei et al. [24] obtained the mechanical and grounding shape representations by conducting ground reaction force and contact strain experiments on the paw pads of domestic cats in various gaits, so as to explore the adaptive adjustment of the mechanical characteristics and shape of the paws in various gaits. Biewener [25] concluded that, during exercise, cats' paw pads can effectively buffer the ground's vertical reaction force that is 2-3 times the value of their body weight. Zhang et al. [26] carried out a theoretical analysis of the paw pads' vibration reduction characteristics according to the changing law of the vertical ground reaction force as the cat fell on the ground and constructed a mass-spring viscoelastic mechanical model. For the bionic research of nonpneumatic tires, a nonpneumatic tire developed by the Madison Polymer Research Center, Wisconsin, USA, uses a bionic honeycomb structure [27], and the hexagonal honeycomb-like structure is recognized in the field of coupled bionics as a structure with good buffering and energy absorption characteristics [28, 29]. Huang et al. [30] took advantage of the silent characteristics of the stripe structure in the feathers of owls to add nonsmooth structural units on the surface of the spokes to reduce the aerodynamic noise of nonpneumatic tires. According to the good shock absorption and buffering characteristics of a kangaroo's lower limb structure, Zhang et al. [31] made a bionic modification design to the spoke structure. They confirmed that the bionic nonpneumatic tire's performance is better than that of a pneumatic tire relative to radial stiffness, lateral stiffness, longitudinal stiffness, torsional stiffness, and tire ground pressure under different loads. An in-depth exploration of bionics' functional characteristics and mechanism could improve its accuracy and effectiveness and its possible application on nonpneumatic tires. Therefore, with the aim of making the extremely strong vibration reduction characteristics of cat's paw pads when in contact with the ground be applied to the spokes of the nonpneumatic tire, it is necessary to conduct research on the vibration reduction mechanism of the cat's paw pad and get an improved method suitable for the spokes.

The article "Research on Vibration Reduction Method of Nonpneumatic Tire Spoke Based on the Mechanical Properties of Domestic cat's Paw Pads" was published in 2021. Journal: Appl Bionics Biomech.

Existing researches on vibration reduction of spokes of nonpneumatic tires are limited to exploring the impact vibration by changing the spokes' structural parameters and the use of materials to find a relatively optimized damping solution. Structural parameters play a limited guiding role for real vehicle applications of nonpneumatic tire development in the future. Hence, this paper conducts grounding mechanical tests on domestic cats' paw pads to analyze how they achieve natural vibration reduction under normal walking gait and applied this bionic concept to modify spoke-type nonpneumatic tire spoke structures. The asymmetric arc design was carried out on both sides of the spokes to achieve a vibration reduction effect similar to that of the domestic cat's paw pads to optimize the tire's radial vibration characteristics. Then, the vibration reduction effect of the asymmetric arc tire and the original tire is compared. With vibration reduction being the optimization goal, the bionic modified optimized parameters of the spokes were achieved by performing optimization analysis relative to other structural parameters to obtain the optimal vibration reduction spoke structure.

## 2. Research on the Vibration Reduction Mechanism of the Paw Pads of Domestic Cats

### 2.1. The Mechanical Test of the Contact between the Paw Pads and the Ground

The purpose of the mechanical test of the contact between the paw pads and the ground is to obtain the paw pads' vertical reaction force and the strain characteristics during the contact and normal walking gait (*v* = 0.4~0.8 m/s) of domestic cats. The test subjects were four healthy, nondefective domestic cats aged between 4 and 7 years, whose weights ranged from 3.8 to 5.6 kg, and having a shoulder height between 20 and 28 cm. The mechanical test site was provided by the Graduate Laboratory of Tire and Vehicle Rubber of Jiangsu University, China.

The article "Research on Vibration Reduction Method of Nonpneumatic Tire Spoke Based on the Mechanical Properties of Domestic cat's Paw Pads" was published in 2021. Journal: Appl Bionics Biomech.

During the test, a pressure-sensitive walkway (Walkway A101; Tekscan, the USA) was used to measure the paw pads' vertical reaction force when the domestic cats walked across the pressure plate in a straight line at different speeds. In order to obtain the strain characteristics of the domestic cats' with the ground, black spots and speckles were applied on their paw pads as they walk straight on the glass plate, as shown in Figure 1(a). A high-speed camera (Olympus i-SPEED 3, Japan) installed under the glass plate was used to record the motion of the paw pads, and then, the images were digitally processed using the VIC-2D of the CSI company in the United States to obtain the strain and related information of the contact between the paw pads and the ground, as shown in Figure 1(b).

### 2.2. The Mechanical Analysis of the Contact between the Paw Pads and the Ground

For each domestic cat, six valid data were taken for processing. Each part's peak vertical ground reaction force is expressed as a percentage of the domestic cat's body weight (%BW); recorded as mean value ± standard deviation. As shown in Figure 2, the domestic cat paw pad is divided into a palm pad and four toe pads; the second, third, fourth, and fifth toe pads, respectively. Peak vertical ground reaction force in each area of the fore and hind paw pads of cats is depicted in Table 1. As shown in Table 1, the peaks of the toe pads and palm pads of the fore paw pads are higher than those of the hind paw pads, and the palm pad area bears the maximum peak value of the entire paw pad area. Accordingly, the palm pad area of the fore paw pads of the cat is the key area for realizing the vibration reduction function.

The main strain field's distribution and the strain directions of the domestic cat's fore paw pad during the whole grounding process are displayed in Figure 3. The *X* and *Y* axes show the paw pad forward and inner directions, respectively. In terms of the principal strain directions, the four toe pads did not change during the whole grounding process (*Y*-oriented tensile deformation). The palm pad area was mainly under tensile strain in the *Y* direction before 0.18 s, and it was primarily in the *X* direction after 0.18 s, which indicated that the palm pad had a swing deformation phenomenon in the contact surface. And the main strain values of the four toe pads' continued to increase during the entire contact process. The palm pad's strain value increased first and then decreased alternately in the inner and outer regions. The palm pad's maximum main strain value was significantly lower than that of the toe pads, which was caused by the change of the strain directions.

The article "Research on Vibration Reduction Method of Nonpneumatic Tire Spoke Based on the Mechanical Properties of Domestic cat's Paw Pads" was published in 2021. Journal: Appl Bionics Biomech.

To further clarify the vibration reduction effect of the palm pad's swing deformation, the variation trends of the strain values in the *X* and *Y* directions of the 3^rd^ toe pad and palm pad during the grounding process are extracted, and the results are depicted in Figure 4. Considering that the incompressibility of the paw pad would cause its local compression in the *X* or *Y* directions to be transformed into a tensile deformation in the *Y* or *X* directions, the strain values greater than zero in the *X* and *Y* directions of the 3^rd^ toe pad and palm pad were averaged to characterize the strain values in the *X* and *Y* directions, and the strain values were recorded as *E*_*x*_ and *E*_*y*_, respectively. It can be seen from Figure 4 that both *E*_*x*_ and *E*_*y*_ of the 3^rd^ toe pad generally show increasing trends as a whole, while the fluctuating changes of the opposite trends of *E*_*x*_ and *E*_*y*_ in the palm pad can achieve the strain attenuation value.

A careful analysis of the toe and palm pads' main strain changing characteristics shows that a vibration-damping effect is realized when the palm pad deformation swings in the *X* and *Y* directions; that is front-rear and left-right swinging deformation.

## 3. Bionic Vibration Reduction Design for Spokes of the Nonpneumatic Tire

The vibration characteristics of tires are an important factor affecting the NVH of vehicles [32]. The vibration source in the nonpneumatic tire during the rolling process is primarily from the buckling and rebound of the spokes under tension when entering and leaving the contact area, the interaction between the discrete spokes and the ring, the interaction when the ring is in contact with the ground, and the force of the ground and the vibration between the ring and the spoke transmitted to the hub [19]. Therefore, the spokes have a great influence on the vibration of nonpneumatic tires. Based on the vibration reduction mechanism of the swing deformation of the domestic cat's paw pads, the spokes can be designed with bionics to improve the vibration characteristics of the nonpneumatic tires and enhance the NVH performance of the vehicle.

### 3.1. Finite Element Simulation Analysis of the Nonpneumatic Tire

#### 3.1.1. The Geometry of the Nonpneumatic Tire

In this paper, Michelin's Tweel nonpneumatic tire (Figure 5) is selected because of its relatively established and wide application. The geometric parameters of Tweel are selected from the research of Bezgam [19]. The structural composition and material usage of the three-dimensional geometric model of the nonpneumatic tire is shown in Figure 6. Tweel is mainly composed of four parts: a rigid hub, deformable spokes, a flexible ring with reinforcements, and a tread. The wheel hub is made of aluminum alloy, which supports the tire and is assembled with the shaft. The spokes are in pairs, the whole wheel consists of 25 pairs of spokes, and the material of the spokes is polyurethane. The flexible ring is divided into three parts by two reinforcements. From the inside to the outsides, there are the inner coverage, the shear layer, and the outer coverage using a polyurethane material. The shear band between the two reinforcements mainly bears the shear force when the tire is rolling under load. The reinforcements are made of high-strength steel, providing high rigidity and strength in the circumferential direction. The tread is made of rubber to ensure that the tire has excellent friction and better road gripping ability,

The article "Research on Vibration Reduction Method of Nonpneumatic Tire Spoke Based on the Mechanical Properties of Domestic cat's Paw Pads" was published in 2021. Journal: Appl Bionics Biomech.

#### 3.1.2. Establishment and Verification of Finite Element Model

The finite element model is displayed in Figure 7. The polyurethane material is modeled using the Marlow model, while the rubber is modeled with the Neo-Hookean model. The specific material properties settings is adopted from [19, 20, 33]. Using the Abaqus/Standard solution method, the road surface is defined as a rigid analytical body and is fixed. A radial force of 3665 N (a quarter of the rated load of the nonpneumatic tire) is applied to the rim's center to simulate the tire grounding process. The Coulomb friction model describes the contact characteristics between the tire and the road surface.

Figure 8 displays the load deflection curve (vertical stiffness curve) between the simulation value of the finite element model and the analysis result of the Akshay Narasimhan curve [21]. The stiffness curves of the two are relatively close, and the error for a radially loaded of 3665 N tire is only 0.97%. The comparison results illustrate that the finite element model established in this paper can accurately reflect the mechanical characteristics of Tweel for further research.

### 3.2. Bionic Design of Spokes

Ramachandran et al. [34] carried out a study on the spoke vibration and concluded that under the same conditions, the vertical middle node vibrates more violently than the upper and lower quarter nodes in the radial direction of the spoke. The vibration gradually increases from the middle position towards the edges on both sides in the axial direction. Therefore, a scallop-shaped treatment method on the side edge of the spokes is proposed: it involves a precise cutting out of the areas with severe vibrations to reduce the vibration amplitude. Figures 9 and 10 show the spoke vibration marker nodes and the scallop-shaped edges, respectively.

The article "Research on Vibration Reduction Method of Nonpneumatic Tire Spoke Based on the Mechanical Properties of Domestic cat's Paw Pads" was published in 2021. Journal: Appl Bionics Biomech.

Inspired by the scallop-shaped spoke edges treatment and the domestic cat's paw pad vibration reduction mechanism, an asymmetric structural design is carried out on the spokes to enable the tire to achieve similar swing deformation characteristics in the rolling process. The bionic modification design is presented in Figure 11. The vertices (*P*) of the asymmetric arc are on the horizontal straight line where the upper and lower quarter nodes are located. The size of the arc is determined by the vertical distance *h*_1_ from the *P* to the connecting line (edge line) of the top and bottom points, which is 15 mm here. The shape of the arc is constructed based on the method of cubic interpolation spline curve. The left-right and up-down swing of the tire during rolling is realized by distributing the arcs asymmetrically at both sides of the spoke to the axial and radial bisecting lines accordingly. And the front-rear swing is also realized by the asymmetric arrangement of the adjacent spokes. In ensuring the stability of tire bearing capacity, the spokes are staggered along the circumferential direction of the tire in accordance with the asymmetric arc of spokes 1 and 2, as displayed in Figure 12. Consequently, the asymmetrical arc not only cuts off a part of the spokes where the vibration is relatively large but also dissipates the impact from the ground in the swing deformation of the spokes to attain the overall vibration reduction effect.

To eliminate the influence of the bionic structural design and to assess the vibration reduction performance of the asymmetric arc swing deformation, a comparison of asymmetric and symmetric arc tires of the same weight is made. As depicted in Figure 13, the *P* of the symmetric arc is on the horizontal line where the vertical middle node is located, and the vertical distance *h*_2_ from the *P* to the edge line represents the size of the symmetric arc, which is 15 mm.

### 3.3. Finite Element Analysis and Discussion of Bionic Design

The vibration and noise of tires are closely related to the radial excitation force of the road surface during rolling, and the larger the excitation force value is, the higher the vibration and noise value will be [32, 35]. With the aid of the Abaqus/Explicit method, the hub, spokes, inner and outer coverages, shear layer, and tread adopt an 8-point linear hexahedral three-dimensional stress element with reduced integration (C3D8R). The reinforcement layer has elements of 4-node and quadrilateral with reduced integration (SFM3D4R). For simulation analysis, a radial load of 3665 N and a speed of 60 km/h are applied to the rim. And the road condition is considered fixed. Then, the radial excitation force of the road in the time domain of 0.12 s (steady rolling 1.06 cycles) when the tire is rolling in a steady state is extracted. The comparison of the radial excitation force of three kinds of tires in the time domain is shown in Figure 14. The radial excitation force of the three types of tires fluctuates up and down at the applied load of 3665 N. The fluctuation of the symmetrical arc tire is the most obvious, followed by the original tire. In contrast, the radial excitation force of the asymmetric arc tire has been reduced, especially at the peak, and the excitation force fluctuates more uniformly in the entire time domain. Therefore, the application of asymmetric arcs on the spokes can significantly reduce the radial vibration of the tire.

The article "Research on Vibration Reduction Method of Nonpneumatic Tire Spoke Based on the Mechanical Properties of Domestic cat's Paw Pads" was published in 2021. Journal: Appl Bionics Biomech.

To further demonstrate that the asymmetric arc tire is superior to both the symmetric arc tire and original tire in vibration reduction and further clarify the reason why asymmetric arc tire can reduce the radial excitation force of the road surface, the FFT function in MATLAB is used to convert the excitation force in the time domain to the amplitude change in the frequency domain. Since the sound pressure level (SPL) with a frequency lower than 100 Hz has no significant effect on human perception of noise [14], and when the frequency is greater than 1500 Hz, the amplitudes are small, and there are no significant peak amplitudes. So 100 Hz-1500 Hz is taken as the range of analysis in this paper.  Figure 15 shows the spectrum comparison between the original tire and the asymmetric arc tire. Figures 15 and 16 , respectively, show the comparison of the spectrum between the original tire and the asymmetric arc tire and the comparison of the asymmetric arc tire and the symmetric arc tire. And the PA^1^ (peak amplitude 1, lower frequency) and PA^2^ (peak amplitude 2, higher frequency) have been marked. Through comparison, it is found that the PA^1^, PA^2^, and amplitudes corresponding to most frequencies in the entire frequency domain of the asymmetric arc tire are smaller than those of the original tire and the symmetric arc tire.

Since the root mean square (RMS) value can reflect the amplitudes of the overall vibration in the entire frequency range, and the peak amplitude reflects the vibration intensity at the local frequency; this paper uses both the root mean square value and the peak amplitude to quantify the amplitudes of the ground response to further clarify the effect of bionic modification of spokes. The comparison of the amplitudes of the three tires is shown in Table 2, and the formula for calculating the root mean square value is defined as

(1) $$\begin{array}{c} \text{RMS}=\sqrt{\frac{1}{N}\overset{N}{\underset{i=1}{\sum }}{\left(x_{i}\right)}^{2},} \end{array}$$

where *N* is the total number of intervals in the step and *x*_*i*_ is the data on the *i*th interval.

The article "Research on Vibration Reduction Method of Nonpneumatic Tire Spoke Based on the Mechanical Properties of Domestic cat's Paw Pads" was published in 2021. Journal: Appl Bionics Biomech.

As can be seen from Table 2 that the peak amplitude and root mean square value of the asymmetric arc tire are significantly reduced compared to the original tire. The PA^1^, PA^2^, and RMS are reduced by 4.98%, 43.23%, and 16.46%, respectively, indicating that the asymmetric arc can effectively reduce the radial vibration of the tire. Although the PA^2^ of the symmetrical arc tire is lower than that of the original tire, the PA^1^ at the low-frequency band that has a greater impact on tire vibration is 35.14% higher than that of the original tire, significantly increasing the local vibration intensity and its RMS is higher than that of the original tire.

In the comparison between the asymmetric arc tire, the symmetric arc tire, and the original tire, it is found that not only does the peak amplitudes of the asymmetric arc tire decrease but also the overall vibration amplitudes decrease. This indicates that the asymmetric arc tire can weaken the impact through the characteristics of swing deformation to achieve a better vibration reduction effect and authenticates the feasibility of bionic vibration reduction.

## 4. Optimization for Vibration Reduction of Spokes

The feasibility of applying the vibration reduction mechanism of cat's paw pad to the spokes of nonpneumatic tires was verified. However, considering that other parameters of the spokes will also have a certain impact on the vibration of the tires, and therefore without changing the inner and outer diameters of the tire (the length of the spokes remains unchanged), the asymmetric arc is combined with the thickness and curvature of the spokes to optimize the design of the spokes to achieve a better damping effect. The specific process of the design optimization of the spokes structure is illustrated in Figure 17.

1. Parameterization: the optimization design include choosing the right design variables and reducing the number of design variables to reduce complications and cost. [36]. The spoke could be parameterized by three variables: the size of the asymmetric arc, the thickness, and the spoke's curvature
2. Design of experiments (DOE) method: the DOE method provides a reasonable and effective method to obtain information and data, which directly affects the quality of the approximation model and is one of the most important statistical methods in the optimization process. Here, the orthogonal array (OA) was chosen to generate the sample points
3. Finite element analysis numerical test: a model database was established based on the DOE method, and ABAQUS simulations were performed on each model. The selection of the model simulation method and the calculation settings remained the same as before
4. Approximate model (AM) method: the AM method is a mathematical model that approximates a set of input variables (independent variables) and output variables (response variables) through a mathematical model. It is established according to the relationship between the design variables and the simulation response. Here, the Kriging model was selected to build an approximate model
5. Optimization calculation: after constructing the approximate model, a reasonable algorithm is used to solve the objective function to obtain the optimal design parameters. In this paper, a genetic algorithm (GA) was employed to obtain the optimal solution

The article "Research on Vibration Reduction Method of Nonpneumatic Tire Spoke Based on the Mechanical Properties of Domestic cat's Paw Pads" was published in 2021. Journal: Appl Bionics Biomech.

### 4.1. Design of Experiments Method

The design of the experiment method can identify key experimental factors, determine the best combination of parameters, analyze the relationship between independent and dependent variables, and provide sample data for constructing an approximate model [37]. In the process of designing the experiment, the design points of the experiment should cover the design space evenly and avoid the repetition of sampling points as far as possible; the number of test analysis should be minimized to ensure that the calculation cost is not too high under the premise of ensuring accuracy. All the above stated practical requirements were satisfied by applying the orthogonal array (OA) method since it considers both the interaction and the test accuracy and delivers an advantage of high efficiency, speed, and economy.

According to the requirement of orthogonality, an OA table in the form of *L*_*n*_(*E*^*P*^) is generated to design the experiment, where *L* is the table, *n* is the total number of design solutions required (the number of rows in the table), *E* is the level of the factors, and *P* is the number of factors. In this experiment, 3 factors and 3 levels were considered, so an orthogonal table of *L*_9_(3^3^) was used.

The three factors of the orthogonal test are the size of the asymmetric arc (*A*), the thickness of the spoke (*B*), and the curvature of the spoke (*C*). The definition of the thickness and curvature of the spoke are shown in Figure 18; *h*_3_ depicts the vertical distance from the vertical middle node to the line connecting the top and bottom nodes. The size of the distance expresses the magnitude of curvature, the thickness of the spoke is represented by*h*_4_, and the size of the asymmetric arc was described in Section 3.2.

The article "Research on Vibration Reduction Method of Nonpneumatic Tire Spoke Based on the Mechanical Properties of Domestic cat's Paw Pads" was published in 2021. Journal: Appl Bionics Biomech.

The original values of the asymmetric arc is 15 mm, while the thickness and curvature of the spoke are 4.2 mm and 8 mm, respectively. The factors and level design of the orthogonal experiment are indicated in Table 3. The orthogonal table generated according to the factors and levels and the simulation results (RMS) of the nine groups of design schemes are shown in Table 4.

As can be seen from Table 4, compared with the original tire, the RMS values of all the nine schemes are reduced, with the smallest and the largest decreasing values being 4.21% and 47.42%; compared with asymmetric arc tires, the RSM values of the four groups of design schemes are reduced. The minimum decrease is 6.44%, and the maximum decrease is 37.06%. The result proves that a proper combination of the size of the asymmetrical arc, thickness, and curvature of the spokes can effectively deliver a better vibration reduction effect.

With the view of ascertaining the influence of design variables on the RMS value and the degree of contribution, a Pareto chart as shown in Figure 19 is drawn. It can be seen from the figure that for a single design parameter, the curvature of the spoke has the greatest influence on the RMS value, with a contribution rate of 31.71%, and the increase of the curvature will increase the RMS value, followed by the size of the asymmetric arc and the thickness of the spoke, whose contribution rates are 8.69% and 3.75%, respectively, and as the size of the asymmetric arc and the thickness of the spoke increase, the RMS values decrease. The nonlinear influence of a single variable on the RMS value is dominant. For example, the contribution of *C*^2^ to the RMS value is about 17.81%, that is, the influence on the RMS value is quadratic.  Figure 20 further illustrates the effect of design variables on the RMS value. As can be seen from Figure 20 that the curve of *C*^2^ has a larger curvature, the trends of the curves of *A* and *B* are more synchronized, which explains that the size of the asymmetrical arc and the thickness of the spoke have a relatively similar effect on the RMS value. In addition, the Pareto chart also provides the correlation between the design variables and the target variables, in which, the correlation between *A* and *B* has the greatest impact on the RMS value; a value of about 18.57%, indicating that both changes have the greatest influence. *A* and *C* have the least influence on the RMS value (about -1.33%).

The article "Research on Vibration Reduction Method of Nonpneumatic Tire Spoke Based on the Mechanical Properties of Domestic cat's Paw Pads" was published in 2021. Journal: Appl Bionics Biomech.

### 4.2. Approximate Model Method

#### 4.2.1. Kriging Approximation Model

Approximate models include the response surface model (RSM), RBF/EBF neural network model, orthogonal polynomial, and Kriging model. However, since RSM model is not capable of describing nonlinear problems, the RBF model takes a long time to build a model, and considering that the problem studied in this paper does not only have a high degree of nonlinearity but also has random errors, the Kriging model was selected for the construction of an approximate model [38]. The Kriging model can be expressed as

(2) $$\begin{array}{c} y\left(x\right)=f\left(x\right)+Z\left(x\right), \end{array}$$

where *y*(*x*) is the unknown deterministic function, *f*(*x*) is a known approximation function, *Z*(*x*) is the realization of a stochastic process with mean zero, variance *σ*^2^, and nonzero covariance *f*(*x*) provides a global approximation model of the design space, and *Z*(*x*) creates localized deviations so that the Kriging model can interpolate the sample points [39]. In many cases, *f*(*x*) is taken as a constant, and *β* is also employed in the design of spokes structure of nonpneumatic tires.

The covariance matrix of *Z*(*x*) is formulated as

(3) $$\begin{array}{c} \mathrm{cov}\left[Z\left(x^{i}\right),Z\left(x^{j}\right)\right]=\sigma^{2}M\left[R\left(x^{i},x^{j}\right)\right], \end{array}$$

where *R*(*x*^*i*^, *x*^*j*^) is the correlation function between any two input points *x*^*i*^ and *x*^*j*^ of *n* observed points, and *M* is the *n* × *n* correlation matrix with values along the diagonal [40]. Gaussian correlation function was used to calculate *R*(*x*^*i*^, *x*^*j*^) and is given by:

(4) $$\begin{array}{c} R\left(x^{i},x^{j}\right)=\exp\left[-\overset{p}{\underset{k=1}{\sum }}\theta_{k}{\left(x_{k}^{i}-x_{k}^{j}\right)}^{2}\right], \end{array}$$

where *x*_*k*_^*i*^ and *x*_*k*_^*j*^ are the *k*th components of sample points, and *θ*_*k*_ are the unknown correlation parameters, which can be obtained by the maximum-likelihood estimation (MLE) [41] method according to

(5) $$\begin{array}{c} \underset{\theta_{k}>0}{\max}\left[\Phi \left(\theta_{k}\right)\right]=-\frac{1}{2}\left(n\ln{\overset{\wedge }{\sigma }}^{2}+\ln\left|M\right|\right). \end{array}$$

While any value for *θ*_*k*_ creates an interpolative Kriging model, the ‘best' Kriging model is found by solving the *k*-dimensional unconstrained nonlinear optimization problem given by equation (5) [42]. For a given *θ*, the closed-form solution for the optimal values of *β* and *σ*^2^ can be obtained and formulated as

(6) $$\begin{array}{c} \hat{\beta }={\left(I^{T}M^{-1}I\right)}^{-1}\left(I^{T}M^{-1}I\right)Y,\\ {\overset{\wedge }{\sigma }}^{2}=\frac{1}{n}{\left(Y-I\overset{\wedge }{\beta }\right)}^{T}M^{-1}\left(Y-I\hat{\beta }\right), \end{array}$$

where *I* is a *d*-dimensional unit vector and *Y* = [*y*(*x*^*i*^), ⋯, *y*(*x*^*m*^)] is the vector of true limit state function values [43].

The article "Research on Vibration Reduction Method of Nonpneumatic Tire Spoke Based on the Mechanical Properties of Domestic cat's Paw Pads" was published in 2021. Journal: Appl Bionics Biomech.

Predicted estimates, *y* at untried values of *x*, are given by

(7) $$\begin{array}{c} \hat{y}\left(x\right)=\hat{\beta }+r^{T}\left(x\right)M^{-1}\left(Y-I\hat{\beta }\right), \end{array}$$

where *r*^*T*^ is the correlation vector given by

(8) $$\begin{array}{c} r^{T}\left(x\right)={\left[R\left(x,x^{1}\right),\cdots ,R\left(x,x^{i}\right)\right]}^{T}\left(i=1,\cdots ,n\right). \end{array}$$

Therefore, the constant term of the Kriging model is used for the global portion, while the Gaussian correlation function (4) is used for the local deviations.

#### 4.2.2. Error Analysis

When constructing the Kriging model, there will be errors caused by the polynomial model itself or fitting. Therefore, the squared multiple correlation coefficient *R*^2^ is introduced to verify the reliability of the Kriging model. The closer *R*^2^ is to 1, the more accurate the fitting will be. The final result shows that *R*^2^ = 0.99, for which, a conclusion can be drawn that, the Kriging model has sufficient accuracy to interpolate these 9 sample points for optimization calculations.

In this case, two groups of variables were randomly selected, and the ABAQUS and Kriging models were, respectively, used to obtain the RSM values. As illustrated in Table 5, the error between the calculation results of the Kriging model and those of ABAQUS is small, which further verifies the accuracy of the Kriging model.

### 4.3. Optimization Calculation

The genetic algorithm (GA) is a global optimization method that mainly uses the laws of biological evolution to solve optimization problems. GA encodes the individuals and then performs the genetic operations of selection, crossover, and mutation on the encoded individual to seek the optimal solution [44]. In this study, the multi-island genetic algorithm (MIGA), which can be regarded as an improved genetic algorithm, was used to solve the optimal solution. MIGA divides a large population into several subpopulations, each of which carries out genetic operations independently, and the individuals on each island transfer to other islands in a certain proportion periodically to complete the periodic exchange of information [42].

Objective constrained optimization problem can be defined as follows:

Objective function: minimize RMS

Design variables with limits:

(i)7.50 ≤ *A* ≤ 22.50

(ii)2.10 ≤ *B* ≤ 6.30

(iii)4.00 ≤ *C* ≤ 12.00

The RMS value was optimized by MIGA. The size of the subpopulation is 100, the number of islands is 100, and the number of evolutionary generations is 10. The optimization result is *A* = 17.31, *B* = 4.85, and *C* = 6.04. The RMS value for the optimization result is 16.30, which is 4.12% better than the optimal value in the OA table. And the optimization values of *A*, *B*, and *C* are reduced by 7.68% and 7.62% and increased by 0.67%, respectively, compared with the design variables of the optimal vibration reduction in the orthogonal experiment. The values of design variables and RMS of the two groups are not much different, which verifies the reliability of the Kriging model from another perspective.

The article "Research on Vibration Reduction Method of Nonpneumatic Tire Spoke Based on the Mechanical Properties of Domestic cat's Paw Pads" was published in 2021. Journal: Appl Bionics Biomech.

The values of optimized design variables are used for simulation analysis and compared with the original tire and the asymmetric arc tire, and the distribution diagram of the radial excitation force of the three is obtained, as depicted in Figure 21. It manifests that although several peaks of the optimized tire are increased, the local fluctuations around the peaks are reduced; and the green markers illustrate that the fluctuation curve is relatively straight, therefore, the fluctuations during the whole cycle are greatly reduced. The spectrum comparison of the three tires is shown in Figure 22, which indicates that the PA^1^ value of the optimized tire is much smaller than that of the original tire and asymmetric arc tire, and the PA^2^ value and RMS value are also significantly reduced. The result of the comparison proves that the optimized tire has a more prominent advantage of vibration reduction.

According to the simulation results, the RMS value of the optimized tire is 15.63, while the value obtained by MIGA is 16.30, with an error of only 4.11%. In addition, since the original tire and the asymmetric arc tire both use the results of simulation calculations, the simulation values of the optimized tire are used for comparative analysis.  Table 6 shows the comparison of the values of PA^1^, PA^2^, and RMS value among the original tire, asymmetric arc tire and optimized tire. Compared with the original tire, the PA^1^, PA^2^, and RMS values of the optimized tire are reduced by 76.07%, 52.88%, and 51.65%, respectively. The values of PA^1^, PA^2^, and RMS of the optimized tire are 74.82%, 17.00%, and 42.13% lower than those of the asymmetric arc tire, respectively. Results show that using the size of the asymmetric arc, the thickness, and curvature of the tire as design variables to optimize the design has an excellent vibration reduction effect. And combined with the comparison of the structural parameters of the asymmetric arc tire and the optimized tire in Table 7, it is found that increasing the size of the asymmetric arc and the thickness of the spoke appropriately and reducing the curvature of the spoke will have a better vibration reduction effect.

The article "Research on Vibration Reduction Method of Nonpneumatic Tire Spoke Based on the Mechanical Properties of Domestic cat's Paw Pads" was published in 2021. Journal: Appl Bionics Biomech.

## 5. Conclusion

In this paper, the spokes of the nonpneumatic tire were treated with asymmetric arc using the vibration reduction mechanism of domestic cat's paw pads, and the vibration characteristics of the asymmetric arc tire, symmetric arc tire, and original tire under rolling conditions were compared and analyzed. Furthermore, the size of the asymmetric arc, the thickness and curvature of spokes were used as design variables for vibration reduction optimization, and the following conclusions were drawn.

1. Using the pressure-sensitive walkway, high-speed camera, and VIC-2D to carry out the grounding mechanical tests of the paw pads of domestic cats, it was found that the peak vertical ground reaction force of the fore paw pad was greater than that of the hind paw pad, and there were significant differences in strain between the four toe pads and the palm pad. The strains in the *X* and *Y* directions of the four toe pads showed a cumulative increasing trend over time, while in the palm rest area, *E*_*x*_ and *E*_*y*_ did not show a trend of increase over time, and each exhibited fluctuating changes and the trends were opposite to each other; in other words, when *E*_*x*_ increases or decreases, *E*_*y*_ correspondingly decreases or increases, which means that the palm pad through front-rear, left-right swing deformation to weaken the ground impact to achieve the purpose of vibration reduction
2. First of all, the finite element model of the spoke-type nonpneumatic tire was established, and its stiffness curve was compared with those in the reference. The small error between the two verified the feasibility of the model. After that, based on the principle of bionics, the spoke structure of the asymmetric arc was proposed. Through the comparative analysis of radial vibration, it was found that the peak amplitude values and root mean square value of the asymmetric arc tire were distinctly lower than those of the symmetric arc tire and original tire, which proved that asymmetric arc tire had significant vibration reduction characteristics. Finally, it can be concluded that the swing deformation vibration reduction mechanism of the cat's paw pads had a positive vibration reduction effect when applied to the spokes of nonpneumatic tires
3. To maximize the vibration reduction performance of the structural design of the spokes, based on the bionic design of the asymmetric arc, an optimization for vibration reduction using the OA method, the Kriging approximate model, and the MIGA was employed to obtain the optimal design parameters of the spokes. The DOE analysis revealed the curvature of the spokes as the most key parameter for vibration reduction, followed by the size of the asymmetric arc and the thickness of the spokes, while increasing the size of the asymmetric arc and the thickness of the spokes and decreasing the curvature of the spokes appropriately will obtain a better vibration reduction effect. Results showed that the optimal combination of the design variables can reduce PA^1^, PA^2^, and RMS values by 74.82%, 17.00%, and 42.13%, respectively, compared with the asymmetric arc tire, and 76.07%, 52.88%, and 51.65% lower than those of the original tire, respectively

The article "Research on Vibration Reduction Method of Nonpneumatic Tire Spoke Based on the Mechanical Properties of Domestic cat's Paw Pads" was published in 2021. Journal: Appl Bionics Biomech.

## Figures and Tables

**Figure 1:** The contact tests of paw pads: (a) contact pressure test and (b) contact strain test.

**Figure 2:** The paw pad of the cat.

**Figure 3:** The contact strain results of fore paw pad (*t*_total_ = 0.300 s).

**Figure 4:** Distribution of strain values in *X* and *Y* directions in the (a) 3^rd^ toe pad area and (b) palm pad area.

**Figure 5:** Early prototype of Tweel.

**Figure 6:** Structural and material compositions of the nonpneumatic tire.

**Figure 7:** Finite element model.

**Figure 8:** Comparison of radial stiffness curve for simulation and Narasimhan analysis value.

**Figure 9:** Vibration marker nodes for spoke.

**Figure 10:** The scallop-shaped treatment on the side edge of the spokes.

**Figure 11:** Bionic modified design of spoke.

**Figure 12:** Asymmetrical arc structure of spoke pair.

**Figure 13:** Symmetrical arc structure of spoke.

**Figure 14:** Comparison of time-domain distribution of radial excitation force of three kinds of tires.

**Figure 15:** The spectrum comparison between the asymmetrical arc tire and the original tire.

**Figure 16:** The spectrum comparison between the asymmetrical arc tire and the symmetric tire.

**Figure 17:** Flowchart of the design optimization

**Figure 18:** The definition of the thickness and curvature of the spoke.

**Figure 19:** Pareto chart for the RMS.

**Figure 20:** Main effect plot for the RMS.

**Figure 21:** Comparison of the distribution of radial excitation force of three tires.

**Figure 22:** The spectrum comparison between the optimized tire, original tire, and asymmetric arc tire.

**Table 1:** Peak vertical ground reaction force in each area of the fore and hind paw pads of cats.

Pads	Peak vertical ground reaction force (%BW)				
	2^nd^ toe pad	3^rd^ toe pad	4^th^ toe pad	5^th^ toe pad	Palm pad
Fore paw pad	10.9 ± 1.3	14.6 ± 2.3	11.7 ± 1.8	8.7 ± 1.1	37.2 ± 4.4
Hind paw pad	8.3 ± 0.9	12.1 ± 1.5	10.2 ± 1.7	3.9 ± 0.6	25.1 ± 3.2

The article "Research on Vibration Reduction Method of Nonpneumatic Tire Spoke Based on the Mechanical Properties of Domestic cat's Paw Pads" was published in 2021. Journal: Appl Bionics Biomech.

**Table 2:** The comparison of vibration amplitudes of three kinds of tires.

Tire type	Amplitude type		
	PA^1^	PA^2^	RMS
Original tire	226.65	77.93	32.33
Asymmetric arc tire	215.37	44.24	27.01
Symmetric arc tire	349.45	63.34	34.97

**Table 3:** Factors and levels of OAs.

Factor	Level (mm)		
	1	2	3
*A*	11.25	15.00	18.75
*B*	3.15	4.20	5.25
*C*	6.00	8.00	10.00

**Table 4:** Schemes for the OA method.

No.	*A*	*B*	*C*	RMS
1	11.25	3.15	6.00	27.38
2	15.00	4.20	6.00	18.38
3	18.75	5.25	6.00	17.00
4	15.00	3.15	8.00	23.06
5	18.75	4.20	8.00	25.27
6	11.25	5.25	8.00	23.55
7	18.75	3.15	10.00	29.33
8	11.25	4.20	10.00	32.07
9	15.00	5.25	10.00	30.79

**Table 5:** Kriging model validation.

Group	*A* (mm)	*B* (mm)	*C* (mm)	Kriging model	ABAQUS	Error (%)
1	13.13	3.68	7	22.37	21.84	2.43%
2	16.88	4.73	9	27.47	26.47	3.78%

**Table 6:** The comparison of amplitudes.

Tire type	Amplitude type		
	PA^1^	PA^2^	RMS
Original tire	226.65	77.93	32.33
Asymmetric arc tire	215.37	44.24	27.01
Optimized tire	54.24	36.72	15.63

**Table 7:** The comparison of spoke parameters.

Tire type	Parameter		
	*A*	*B*	*C*
Asymmetric arc tire	15 mm	4.2 mm	8 mm
Optimized tire	17.31 mm	4.85 mm	6.04 mm
Increase or decrease	↑15.40%	↑15.48%	↓24.50%

## Data Availability

The data used to support the findings of this study are available from the corresponding author upon request.
